# Segmentation of Breast Tubules in H&E Images Based on a DKS-DoubleU-Net Model

**DOI:** 10.1155/2022/2961610

**Published:** 2022-09-30

**Authors:** Yuli Chen, Yao Zhou, Guoping Chen, Yuchuan Guo, Yanquan Lv, Miao Ma, Zhao Pei, Zengguo Sun

**Affiliations:** ^1^School of Computer Science, Shaanxi Normal University, Xi'an, China; ^2^Shandong Junteng Medical Technology Co., LTD, China

## Abstract

The formation of breast tubules plays an important role in the pathological grading of breast cancer. Breast tubules surrounded by a large number of epithelial cells are located in the subcutaneous tissue of the chest. The shapes of breast tubules are various, including tubular, round, and oval, which makes the process of breast tubule segmentation a difficult task. Deep learning technology, capable of learning complex data structures via efficient representation, could help pathologists accurately detect breast tubules in hematoxylin and eosin (H&E) stained images. In this paper, we propose a deep learning model named DKS-DoubleU-Net to accurately segment breast tubules with complex appearances in H&E images. The proposed DKS-DoubleU-Net model suggests using a DenseNet module as the encoder of the second subnetwork of DoubleU-Net, which utilizes dense features between layers and strengthens the propagation of features extracted in all previous layers, in order to better discover the intrinsic characteristics of breast tubules with complex structures and diverse shapes. Moreover, a feature fusing module called Kernel Selecting Module (KSM) is inserted before each output layer of the two U-Net branches of the DoubleU-Net, to implement a multiscale feature fusion via a self-adaptive kernel selecting for the sake of accurate segmentation of breast tubules in different sizes. The experiments on the public BRACS dataset and a private clinical dataset have shown that our model achieves better segmentation performance, compared to the state-of-art models of U-Net, DoubleU-Net, ResUnet++, HRNet, and DeepLabV3+. Specifically, on the public BRACS dataset, our method produced an F1-Score of 92.98%, which outperforms the F1-Score of U-Net, DoubleU-Net, and HRNet by 4.24%, 0.37%, and 1.68%, respectively, and is much better than performances of DeepLabV3+ and ResUnet++ by 7.83% and 23.84%, respectively. On the private clinic dataset, the proposed model achieved an F1-Score of 73.13%, which has shown an improvement of 10.31%, 1.89%, 4.88%, 15.47%, and 31.1% to the performances of the U-Net, DoubleU-Net, HRNet, DeepLabV3+, and ResUnet++, respectively. Superior performance could also be observed when comparing the proposed DKS-DoubleU-Net with the others using the metrics of Dice and mIou.

## 1. Introduction

Breast cancer is one of the most common cancers for women in the world [1]. With the increase of breast cancer patients worldwide, the precise diagnosis and prognosis of breast cancer have become urgent tasks. The Nottingham grading system [2] has become the most adopted clinic routine criteria in the diagnosis and prognosis of breast cancer. As one of the three essential factors (tubule formation, nuclear pleomorphism, and mitotic counts) in the Nottingham grading system, the assessment of breast tubule formation plays an important role [2].

The arrangement and morphology of tumor cells within breast tubules are vital criterions for the diagnosis of breast ductal carcinoma. Breast ductal carcinoma will destroy the function of breast ducts, resulting in the disappearance of tubular structure of breast tubules. Therefore, it is particularly important to accurately identify breast tubules in pathological images for a precise grading and diagnosis of breast cancer patients.

The identification of breast tubules is usually done by the manual observation of pathologists through microscopes. This process is not only time- and labor-consuming but also prone to errors due to interobserver and intraobserver discrepancies. Thus, it is necessary to develop a model to automatically recognize the breast tubule in histopathological images for a more objective and accurate computational pathology analysis.

Breast tubules are located in the subcutaneous tissue of the chest. Although breast tubules are characterized by clear lumina surrounded by epithelial cells, they are easily confused with clefts induced by shrinkage artifacts [2]. Moreover, breast tubules are typical of diverse appearances, complex structures, and highly sophisticated morphology, such as various shapes (tubular, round, or oval), colors, and textures, as shown in Figure 1. Therefore, it is a challenging task for traditional machine learning methods to identify breast tubules effectively. A promising way is to train end-to-end deep learning models [3–7], which could automatically discover the essential characteristics of breast tubules through the nonlinear representation of multiple layers of neurons.

Nowadays, with the rapid development of deep learning technology, increasing image segmentation models, such as U-Net [8], ResUNet++ [9], DeepLabV3+ [10], DoubleU-Net [11], and HRNet [12], have shown good performance in the field of medical image segmentation. For example, the U-Net model was applied to the segmentation of neuronal structures in electron microscopic recordings and the cell segmentation task in light microscopic images. Moreover, many U-Net-based Convolutional Neural Networks (CNNs) have also demonstrated superior performance in the task of medical image segmentation [13–17]. Particularly, among the outstanding U-Net derived models, DoubleU-Net has shown promising results on various medical image datasets, including polyp detection dataset, lesion boundary segmentation dataset, and nuclei image dataset.

There have been some approaches dedicated to semantically segmenting breast tubules in hematoxylin and eosin (H&E) stained images. For example, Wang et al. [18] proposed a two-step clustering and random forest method for automatic recognition and segmentation of breast tubules. Basavanhally et al. [19] applied the O'Callaghan neighborhood in modeling and imposed spatial distance with directional constraints on object attributes for tubular identification on histopathological images stained with hematoxylin and eosin (H&E). Maqlin et al. [20] used K-means clustering to identify objects including glandular tubules and fatty regions. Zhang et al. [21] proposed a method for detecting tubules in testicular images based on boundary weighting and circular shortest path. Janowczyk and Madabhushi [22] detected breast tubules, lymphocytes, and epithelial cells by using the deep learning framework of the Caffe AlexNet network model.

However, the current deep learning models are still incapable of accurate segmentation of breast tubules, because breast tubules are usually of diverse appearance, complex structures, and different sizes for patients in different grading stages and various tissue transections.

Although deep-learning-based methods have been applied to the segmentation of breast tubules [8–12], most of them have not taken into account the reuse and fusion of multilevel features to better describe the tubule ROI regions of complex structures, diverse shapes, and different sizes for a more accurate segmentation performance.

In this paper, we propose a novel semantic segmentation model named DKS-DoubleU-Net by integrating a DenseNet [23] module and a Kernel Selecting Module (KSM) [24] into the DoubleU-Net model for accurate segmentation of breast tubules in H&E images. The adopted DenseNet encoder utilizes dense features between layers to discover intrinsic characteristics and strengthen the feature propagation of breast tubules. Besides, the KSM module conducts a self-adaptive kernel selecting for the sake of a multilevel feature fusion, facilitating the detection of breast tubules of different sizes. Experiments on the public BRACS dataset [25] and a private clinical dataset have demonstrated the outperformance of the proposed DKS-DoubleU-Net in the semantic segmentation of the breast tubules, compared to the original DoubleU-Net as well as the state-of-the-art segmentation models including U-Net [8], HRNet [12], DeepLabV3+ [10], and ResUNet++ [9].

## 2. Methods

### 2.1. The Proposed DKS-DoubleU-Net Architecture

For accurate semantic segmentation of breast tubules with complex structures and shapes, the proposed DKS-DoubleU-Net model is constructed through two main processes: (1) substituting the encoder of the second U-Net subnetwork branch of DoubleU-Net with a DenseNet [23] module; (2) inserting a Kernel Selecting Module (KSM) before each output layer of the two U-Net branches of the DoubleU-Net. The overall architecture of the proposed DKS-DoubleU-Net model is shown in Figure 2.

As shown in Figure 2, the proposed DKS-DoubleU-Net is composed of two U-Net subnetwork branches which are connected end to end, and each network branch is composed of an encoder and a decoder. Specifically, the VGG19 [26] is employed as the encoder module in the first network branch. The decoder modules of the two subnetwork branches are identical, both including four decoder blocks, and each of the decoder blocks consists of a squeeze and excitement block [27], 3 × 3 convolutional layers, and an upsampling layer. For each branch, the encoder and the decoder are connected with an Atrous Spatial Pyramid Pooling (ASPP) [10], which expands the receptive field of the convolutional layer. When the input image is fed to the first network, a preliminary binary segmentation mask will be generated to indicate the coarse detected regions of the tubules. Subsequently, the binary preliminary output tubule segmentation mask is multiplied by the original input image to remain only the coarse tubule ROI region in the original image. And the coarse tubule ROI image is further served as the input of the second network branch. The KSM module is inserted before each output layer of the two U-Net subnetwork branches. Finally, after the DenseNet encoder module and the decoder block of the second subnetwork branch, the final result of breast tubule segmentation on the input H&E image is output.

We will describe each component of the proposed DKS-DoubleU-Net model in detail.

### 2.2. Encoder

Feature extraction is the major function of the encoders in both branches [28]. The encoder of the first network branch adopts a VGG19 module, and all the convolutional layers of the module employ the same small size of 3 × 3 convolution kernels. Thus, VGG19 with a deep enough network structure could extract plenty of nonlinear features.

As the encoder of the second network branch, the DenseNet with a dense connection mechanism is introduced to extract the complex tubule structure features for a better tubule segmentation in H&E images. Specifically, each Dense Block (as shown in Figure 2(b)) of the introduced DenseNet module densely collects the output feature maps of all previous Dense Blocks as its input. Such dense connection of Dense Blocks makes the propagation and utilization of multilevel features more effective, resulting in a more efficient training process. That is, by establishing dense connections between the front and back layers, the reuse and propagation of features between different layers could alleviate the problem of gradient disappearance caused by the deepening of the network to a certain extent. Therefore, the introduced DenseNet encoder has the potential to effectively extract, fuse, and propagate multilevel features of breast tubules on the ROI regions detected by the first U-Net branch.

### 2.3. Decoder

Decoders are used to restore the feature maps to the original resolution. The model has two decoders, each of which consists of four decoder blocks, as shown in Figure 2(a). For each layer of the decoder block, an upsampling operation is applied to enlarge the image through interpolation [29]. And then the upsampling feature map is concatenated with the feature map output from the corresponding encoder through a skip connection. Different from the skip connection from the encoder to the decoder in the first subnetwork branch, there are two skip connections from both encoder1 and encoder2 to the decoder in the second subnetwork branch. The purpose of this process is to reduce information loss in the process of feature extraction. After the upsampling, there are two 3 × 3 convolution operations, each of which is followed by the operations of normalization and ReLU [30]. The subsequent layers are composed of a squeeze and excitation block, a 1 × 1 convolution operation, and a sigmoid activation function [31]. The final output of the model is a binary image [32] having the same size as the input image to indicate the segmentation regions of breast tubules.

### 2.4. Kernel Selecting Module (KSM)

The Kernel Selecting Module (KSM) fuses multiple convolutional branches with different kernel sizes to implement adaptive receptive field selection and multiscale feature fusion, as shown in Figure 2(c). Firstly, the input *U* ∈ *ℜ*^*H*×*W*×*C*^ performs 3 × 3, 5 × 5, and 7 × 7 convolution operations, respectively, to obtain *U*′ ∈ *ℜ*^*H*×*W*×*C*^, *U*′′ ∈ *ℜ*^*H*×*W*×*C*^, and *U*′′′ ∈ *ℜ*^*H*×*W*×*C*^. Secondly, *U*′, *U*′′, and *U*′′′ are added to obtain $\bar{U}$. The calculation formula of $\bar{U}$ is

(1) $$\begin{array}{c} \bar{U}=U^{\prime }+U^{\prime \prime }+U^{\prime \prime \prime }. \end{array}$$

Then, the global average pooling operation (GAP) and the full connection operation (*FC*_1_) are performed on $\bar{U}$, and after that, we perform the full connection operation (*FC*_2_) on the obtained result again. The specific calculation formula is as follows:

(2) $$\begin{array}{c} \alpha^{\prime }={{FC}_{2}}^{\prime }\left({FC}_{1}\left(GAP\left(\bar{U}\right)\right)\right),\\ \beta^{\prime }={{FC}_{2}}^{\prime \prime }\left({FC}_{1}\left(GAP\left(\bar{U}\right)\right)\right),\\ \gamma^{\prime }={{FC}_{2}}^{\prime \prime \prime }\left({FC}_{1}\left(GAP\left(\bar{U}\right)\right)\right), \end{array}$$

where *α*′ ∈ *ℜ*^1×1×*C*^, *β*′ ∈ *ℜ*^1×1×*C*^, and *γ*′ ∈ *ℜ*^1×1×*C*^. Three obtained outputs are calculated by softmax, respectively. The specific calculation method is as follows:

(3) $$\begin{array}{c} \alpha_{c}=\frac{e^{\alpha_{c}^{\prime }}}{e^{\alpha_{c}^{\prime }}+e^{\beta_{c}^{\prime }}+e^{\gamma_{c}^{\prime }}},\\ \beta_{c}=\frac{e^{\beta_{c}^{\prime }}}{e^{\alpha_{c}^{\prime }}+e^{\beta_{c}^{\prime }}+e^{\gamma_{c}^{\prime }}},\\ \gamma_{c}=\frac{e^{\gamma_{c}^{\prime }}}{e^{\alpha_{c}^{\prime }}+e^{\beta_{c}^{\prime }}+e^{\gamma_{c}^{\prime }}}, \end{array}$$

where *α*, *β*, and *γ* denote the soft attention vectors, respectively. Note that *α*_*c*_ is the *c*-th element of *α*, and is the same for *β*_*c*_ and *γ*_*c*_.

Finally, the feature maps obtained by different convolution kernels and the obtained attention vectors are multiplied and added to obtain the final output feature map *V*.

(4) $$\begin{array}{c} V_{c}=\alpha_{c}\cdot U^{\prime }+\beta_{c}\cdot U^{\prime \prime }+\gamma_{c}\cdot U^{\prime \prime \prime }, \end{array}$$

where *α*, *β*, and *γ* need to satisfy *α*_*c*_ + *β*_*c*_ + *λ*_*c*_ = 1, and *V*=[*V*_1_, *V*_2_, . ⋯ , *V*_*c*_], *V*_*c*_ ∈ *ℜ*^*H*×*W*^.

## 3. Experiments

### 3.1. Datasets

In the task of breast tubule segmentation, we conducted experiments on the public BRACS dataset [25] and a private clinical dataset. For each dataset, we randomly selected 10% of images for testing, 10% of images for verification, and the rest 80% of the images for model training.

The first experimental dataset is a private clinical dataset with a total of 398 images, each of which is 2000 × 2000 in size. The tubule masks on each of the images in this dataset were annotated by a pathologist, with white areas representing the breast tubules and black areas indicating irrelevant areas.

The second dataset is an openly accessible dataset named BRACS, which has a total of 4539 H&E images of various sizes. Since the breast tubules on the images of this dataset were not labeled, we did manual annotation of the breast tubules with the help of a pathologist before our experiments.

### 3.2. Implementation Details

Our experiments ran on the Ubuntu operation system with GPUs of GeForce GTX 1080 [33]. Our model was built using the Keras framework with TensorFlow [34, 35] as the back end. We used the Dice function [36] as the loss function of model training, the optimizer was Adam [37], the learning rate was set to 1e-5, the batch size of the DKS-DoubleU-Net model and those of the other comparable models were set to 4, and the epoch was set to 200.

Our private dataset includes 398 original images with a size of 2000 × 2000 cropped from WSI images and their corresponding ground truths of tubule masks. Since the size of each of the private clinical pictures is 2000 × 2000, to reduce the computational pressure of the graphics processing system [38] and improve the efficiency of code running, we cut each 2000 × 2000 image into 16 random overlapping 512 × 512 tiles, resulting in 6368 tiles in total. Since the cropped images do not change the structures of tubules, it will not affect the actual segmentation effects.

The public BRACS dataset is composed of 4539 H&E images of different image sizes, we resized the images to 512 × 512 for consistency with the 512 × 512 tile size of the private dataset. Since there are no tubule annotations in the public dataset, we generated the labels of the breast tubules beforehand. To speed up the annotation process, we adopted a coarse-to-fine annotation procedure on this dataset.

Specifically, as the first step, we randomly selected 200 H&E images and asked a pathologist to manually annotate the breast tubules using HistoView [39]. Subsequently, we trained the proposed model by using the 200 annotated images and obtained a preliminary model. The preliminary model in our experiment was a DoubleU-Net adopting a deep Residual module as the encoder of the second subnetwork. With the help of this preliminarily trained model, we tested the remaining unlabeled images and treat their outputs as coarse annotations of tubules. Then, the coarse annotations were denoised by applying the “bwareaopen” function in MATLAB to remove small areas [40]. Finally, the refined breast tubule annotations were generated by manually eliminating the false positives and false negatives on the coarse annotation images with the help of the pathologist [41].

### 3.3. The Objective Function and Evaluation Metrics

To train the proposed DKS-DoubleU-Net model, Dice function is used as the loss function to emphasize the accurate semantic segmentation of the tubule regions. The Dice loss function is widely used in medical image segmentation tasks. The definition of Dice Loss is as follows:

(5) $$\begin{array}{c} \text{DiceLoss}=1-\frac{2\left|X\cap Y\right|}{\left|X\right|+\left|Y\right|}, \end{array}$$

where *X*∩*Y* denotes the intersection between *X* and *Y*, |*X*| and |*Y*| represent the number of elements, respectively, and the numerator is multiplied by 2 to ensure that the value range is between 0 and 1.

To measure the superiority of the proposed model more quantitatively and comprehensively, Dice, mIou, Precision, Recall, and F1-Score, which are the most important and commonly used metrics in semantic segmentation tasks [42–45], served as evaluation metrics in our experiments:

(6) $$\begin{array}{c} \text{Dice}=\frac{2\left|X\cap Y\right|}{\left|X\right|+\left|Y\right|},\\ \text{mIou}=\frac{\text{TP}}{\text{TP}+\text{FP}+\text{FN}},\\ \text{Precision}=\frac{\text{TP}}{\text{TP}+\text{FN}},\\ F1-\text{Score}=\frac{2\times \text{Precision}\times \text{Recall}}{\text{Precision}+\text{Recall}}, \end{array}$$

where TP represents true positive, FP denotes false positive, and FN means false negative.

## 4. Results and Analysis

To evaluate the performance of the proposed DKS-DoubleU-Net model, we conducted experiments on both the private clinical dataset and the public BRACS dataset independently. The experiment results of the proposed DKS-DoubleU-Net model are compared with those of the state-of-the-art segmentation models, including U-Net [8], DoubleU-Net [11], ResUnet++ [9], DeepLabV3+ [10], and HRNet [12] models. To assess the performances of different models objectively, we employ the most commonly used evaluation metrics in semantic segmentation tasks, such as Dice, mIou, Precision, Recall, and F1-Score in our experiments.

### 4.1. Experiments on the Private Clinical Dataset

The quantitative comparison of the tubule segmentation results obtained by different models on the private clinical dataset is shown in Table 1. The proposed DKS-DoubleU-Net model achieves a Dice of 70.02%, a mIou of 55.47%, a Recall of 76.36%, a Precision of 70.16%, and an F1-Score of 73.13%, which is superior to the original DoubleU-Net model by increasing 2.04%, 2.39%, 1.86%, 1.91%, and 1.89%, respectively. The individual combination of the DenseNet module or KSM module with the original DoubleU-Net also exhibited an improvement in performance as shown in Table 1. This may be attributed to the combined action of the powerful feature extraction ability of DenseNet and the multiscale feature fusion mechanism of KSM. The former could accurately identify the various shapes of tubules and the latter improves the detection accuracy of tubules in different sizes. Moreover, compared to the U-Net model, the proposed DKS-DoubleU-Net has improved the scores of Dice, mIou, Recall, Precision, and F1-Score obtained by 8.87%, 10.28%, 10.68%, 9.96%, and 10.31%, respectively. In summary, the proposed DKS-DoubleU-Net model has achieved the highest scores in Dice, mIou, and F1-Score, except for precision, among all listed state-of-the-art models. Although the model of “DoubleU-Net+KSM” has the highest precision score, the decrease in its recall score leads to a decrease in its F1-Score (i.e., the harmonic mean of Recall and Precision).

To visualize the performances of different models, we demonstrate several tubule semantic segmentation results on the test set of the private clinical dataset, as shown in Figure 3. As can be seen from Figure 3, DKS-DoubleU-Net has the most excellent performance even in segmenting the challenging targets. Specifically, its segmentation results are the closest to the ground truth images and with the fewest noise spots.

### 4.2. Experiments on the Public BRACS Dataset

To further analyze the performance of breast tubule segmentation by the proposed DKS-DoubleU-Net, we conducted experiments on the public BRACS dataset [25]. The comparative evaluation results of different models on the public BRACS dataset are shown in Table 2.

Table 2 shows that the proposed DKS-DoubleU-Net achieves scores of 92.72% in Dice, 86.55% in mIou, 92.92% in Recall, 93.05% in Precision, and 92.98% in F1-Score. Specifically, after introducing the modules of DenseNet and KSM into the original DoubleU-Net model, the segmentation results have increased by 0.53%, 0.85%, 0.88%, and 0.37% in Dice, mIou, Recall, and F1-Score, respectively. This may be put down to the flexible ability of the introduced DenseNet and KSM modules in segmenting the breast tubules in different sizes and diverse shapes. Compared to the U-Net, the proposed DKS-DoubleU-Net has gained the biggest increase in Dice, mIou, Recall, Precision, and F1-Score by 4.79%, 7.68%, 0.53%, 7.68%, and 4.24%, respectively. On the public BRACS data set, our model fails to reach the highest recall and precision scores, but its F1-Score, resulting from the harmonic mean of recall and precision, is the most superior among all state-of-the-art methods as shown in Table 2.

The illustrative tubule segmentation results obtained by different models on the test set of the public BRACS dataset are shown in Figure 4. It can be seen from Figure 4 that, compared to the state-of-the-art networks, the tubule segmentation results performed by the proposed DKS-DoubleU-Net are more effective in suppressing noisy spots and more accurate in detecting the tubules with various sizes and diverse shapes.

In summary, the proposed DKS-DoubleU-Net model has shown outstanding performance in detecting breast tubules of diverse shapes and different sizes on both the private clinical dataset and the public BRACS dataset.

Specifically, from the quantitative comparison results in Table 1 and Table 2, it can be seen that, among the state-of-the-art models, the proposed DKS-DoubleU-Net model achieves the highest evaluation scores of Dice, mIou, and F1-Score in the tubule segmentation on both datasets. Besides, the compared illustrative tubule segmentation results, as shown in Figures 3 and 4, also demonstrate that the proposed DKS-DoubleU-Net performs best in the accurate breast tubule segmentation, with the results closest to the ground truth among all stat-of-the-art models including DoubleU-Net, U-Net, ResUnet++, DeepLabV3+, and HRNet. Therefore, the introduced modules of DenseNet and Kernel Selecting Module (KSM) in the proposed DKS-DoubleU-Net model could effectively improve the model's ability in complex feature extraction and multiscale feature fusion, which are important in the performance promotion of breast tubule segmentation.

### 4.3. Computational Complexity Analysis

In order to compare the computational complexity of the models, we measure the computational complexity from the amount of parameters (Paras) and the amount of calculation (FLOPs) as shown in Table 3. Each parameter is a float, that is, a parameter is 4 bytes. And the units of these two metrics are MB. The amount of parameters corresponds to the space complexity of the model, that is, the size of the model. The amount of computation corresponds to the time complexity of the model, that is, the length of the network execution time. It can be seen from Table 3 that the amounts of parameters and calculation of the DKS-DoubleU-Net network are a little bit larger than those of the original DoubleU-Net model, due to the addition of the DenseNet and KSM modules. Although the space complexity and time complexity of the DKS-DoubleU-Net network is a little bit higher, it results in a high performance.

## 5. Discussion

Breast tubule formation is one of the three essential factors in the clinical routine Nottingham grading system. The assessment of breast tubule formation is critical to the accurate diagnosis and prognosis of breast cancer [2]. In practice, it is a challenging task to accurately segment the breast tubules in H&E images due to their diverse appearance, complex structures, and highly sophisticated morphology. Although deep-learning-based methods have been applied to the segmentation of breast tubules, most of them have not taken into account the reuse of dense features among layers and the fusion of multilevel features for a more accurate semantic segmentation performance of breast tubules. To solve this problem, the proposed DKS-DoubleU-Net model introduced a DenseNet [23] as the encoder module of the second network branch in DoubleU-Net. Besides, the Kernel Selecting Module (KSM) was inserted in front of the outputs of the two U-Net branches in the proposed DKS-DoubleU-Net.

The potential roles of the two modules played in the task of tubule segmentation could be inferred as follows: (1) the DenseNet module, utilizing dense connections between layers through Dense Blocks, would help better extract features from the tubules with complex structures and diverse shapes and (2) the KMS module, enabling a self-adaptive kernel selecting for feature fusion, would facilitate the discovery of tubules of different sizes. Therefore, both qualitative and quantitative experiments have shown that our model achieves competitive performance on both the private clinical dataset and public BRACS dataset. Specifically, in view of quantitative assessment, the DKS-DoubleU-Net produced a Dice of 70.02% and an F1-Score of 73.13% on the private data, which has increased by 2.04% in Dice and 1.89% in F1-Score compared to the original DoubleU-Net. On the public BRACS dataset, our proposed model achieved a Dice of 92.72% and an F1-Score of 92.98%, which outperformed the DoubleU-Net by 0.53% and 0.37%, respectively. Both in terms of quantitative metrics and qualitative visual perception of the tubule segmentation results, our model showed the best performance among the state-of-the-art models, including DoubleU-Net [11], U-Net [8], ResUnet++ [9], DeepLabV3+ [10], and HRNet [12].

The limitation of the DKS-DoubleU-Net is that after the introduction of DenseNet and Kernel Selecting Module (KSM), the network structure becomes more complex and has more parameters to learn, therefore, in our future work, we will focus on optimizing the network structure for more efficient and accurate segmentation performance on diverse tubule regions. As another limitation, our network cannot handle images of random size. In our experiment, we cropped or resize the input image to the size of 512 × 512. Therefore, to develop an algorithm dealing with input images of random sizes will be one of our further works.

## 6. Conclusions

In this paper, we proposed a semantic segmentation model termed DKS-DoubleU-Net for accurate semantic segmentation of breast tubules in H&E images. The proposed DKS-DoubleU-Net adopted a DenseNet module as the second encoder of the DoubleU-Net and inserted a Kernel Selecting Module (KSM) before the output layer in each of the two U-Net branches. Our purpose is to discover, reuse, fuse, and propagate the dense features and multilevel features extracted from the coarse breast tubular regions suggested by the first U-Net subnetwork branch of DoubleU-Net. Moreover, in the experiment section, we applied the proposed DKS-DoubleU-Net to two datasets. In terms of both quantitative evaluation and visual perception quality, the proposed DKS-DoubleU-Net achieved competitive performance in the semantic segmentation of breast tubules in the H&E images on both datasets, as compared with the state-of-the-art models. Therefore, DKS-DoubleU-Net has the potential of being a baseline for breast tubule segmentation in H&E images.

## Figures and Tables

**Figure 1:** Demostration of the complexity of breast tubules. Breast tubules are usually of diverse appearances, complex structures, and highly sophisticated morphology. The first and third row show several breast tubular images from public BRACS dataset and private clinical dataset. The second and fourth row represent their corresponding ground truths.

**Figure 2:** The overall architecture of the proposed DKS-DoubleU-Net model and the details of the introduced DenseNet and Kernel Selecting Module (KSM) for semantic breast tubule segmentation. (a) The overall architecture of the proposed DKS-DoubleU-Net model. (b) The detailed architecture of the DenseNet module [23]. (c) The detailed architecture of the Kernel Selecting Module (KSM) module [24].

**Figure 3:** The illustrative tubule segmentation results of different models on the test set of the private clinical dataset. The first row lists the original images; images a(1)-f(1) in the second row are the corresponding tubule annotation masks; images a(2)-f(2) in the third row are the tubule segmentation results performed by DKS-DoubleU-Net; images a(3)-f(3) in the fourth row are the results output by the DoubleU-Net which added DenseNet; images a(4)-f(4) in the fifth row are the results obtained by the DoubleU-Net which added Kernel Selecting Module (KSM); images a(5)-f(5) in the sixth row are the results output by the DoubleU-Net; images a(6)-f(6) in the seventh row are the results output by Unet; images a(7)-f(7) correspond to the results of ResUnet++; images a(8)-f(8) are the results obtained by DeepLabV3+, and images a(9)-f(9) show the tubule segmentation results of HRNet.

**Figure 4:** The illustrative tubule segmentation results of different models on the test set of the public BRACS dataset. The first row lists the original images; images a(1)-f(1) in the second row are the corresponding tubule annotation masks; images a(2)-f(2) in the third row are the tubule segmentation results performed by DKS-DoubleU-Net; images a(3)-f(3) in the fourth row are the results output by the DoubleU-Net which added DenseNet; images a(4)-f(4) in the fifth row are the results output by the DoubleU-Net which added Kernel Selecting Module (KSM); images a(5)-f(5) in the sixth row are the results output by the DoubleU-Net; images a(6)-f(6) in the seventh row are the results output by Unet; images a(7)-f(7) correspond to the results of ResUnet++; images a(8)-f(8) are the results obtained by DeepLabV3+, and images a(9)-f(9) show the tubule segmentation results of HRNet.

**Table 1:** The quantitative comparison of the tubule segmentation results obtained by different models on the test set of the private clinical dataset.

Model	Dice	mIou	Recall	Precision	F1-score
DKS-DoubleU-Net	0.7002	0.5547	0.7636	0.7016	0.7313
DoubleU-Net+DenseNet	0.6897	0.5412	0.7442	0.7066	0.7249
DoubleU-Net+KSM	0.6820	0.5364	0.7165	0.7243	0.7204
DoubleU-Net	0.6798	0.5308	0.7450	0.6825	0.7124
U-Net	0.6115	0.4519	0.6568	0.6020	0.6282
ResNet++	0.3922	0.2672	0.6610	0.3081	0.4203
DeepLabV3+	0.5513	0.3955	0.5885	0.5651	0.5766
HRNet	0.6608	0.5085	0.6496	0.7188	0.6825

**Table 2:** The quantitative comparison of tubule segmentation results obtained by different models on the test set of the public BRACS dataset.

Model	Dice	mIou	Recall	Precision	F1-Score
DKS-DoubleU-Net	0.9272	0.8655	0.9292	0.9305	0.9298
DoubleU-Net+DenseNet	0.9247	0.8617	0.9288	0.9259	0.9273
DoubleU-Net+KSM	0.9269	0.8655	0.9328	0.9264	0.9296
DoubleU-Net	0.9219	0.8570	0.9204	0.9319	0.9261
U-Net	0.8793	0.7887	0.9239	0.8537	0.8874
ResNet++	0.6547	0.5020	0.7450	0.6450	0.6914
DeepLabV3+	0.8413	0.7301	0.8547	0.8483	0.8515
HRNet	0.9089	0.8348	0.9368	0.8903	0.9130

**Table 3:** Comparison of the computational complexity of the models.

Model	Trainable params	FLOPs
DKS-DoubleU-Net	127.38 M	254.71 M
DoubleU-Net+DenseNet	127.24 M	254.42 M
DoubleU-Net+KSM	111.88 M	223.69 M
DoubleU-Net	111.73 M	223.40 M
U-Net	98.68 M	197.31 M
ResNet++	15.50 M	30.97 M
DeepLabV3+	155.88 M	311.76 M
HRNet	108.93 M	217.85 M

## Data Availability

The data that support the findings of this study are available from the corresponding author upon reasonable request.
